The article "Genetic algorithm optimized node deployment in IEEE 802.15.4 potato and wheat crop monitoring infrastructure" was published in 2021. Journal: Sci Rep.

# Genetic algorithm optimized node deployment in IEEE 802.15.4 potato and wheat crop monitoring infrastructure

**DOI:** 10.1038/s41598-021-86462-1

**Published:** 2021-04-15

**Authors:** Pankaj Pal, Rashmi Priya Sharma, Sachin Tripathi, Chiranjeev Kumar, Dharavath Ramesh

**Affiliations:** Indian Institute of Technology, Indian School of Mines (IIT-ISM), Dhanbad, Jharkhand 826004 India

**Keywords:** Environmental impact, Electrical and electronic engineering

## Abstract

This proposal investigates the effect of vegetation height and density on received signal strength between two sensor nodes communicating under IEEE 802.15.4 wireless standard. With the aim of investigating the path loss coefficient of 2.4 GHz radio signal in an IEEE 802.15.4 precision agriculture monitoring infrastructure, measurement campaigns were carried out in different growing stages of potato and wheat crops. Experimental observations indicate that initial node deployment in the wheat crop experiences network dis-connectivity due to increased signal attenuation, which is due to the growth of wheat vegetation height and density in the grain-filling and physical-maturity periods. An empirical measurement-based path loss model is formulated to identify the received signal strength in different crop growth stages. Further, a NSGA-II multi-objective evolutionary computation is performed to generate initial node deployment and is optimized over increased coverage, reduced over-coverage, and received signal strength. The results show the development of a reliable wireless sensor network infrastructure for wheat crop monitoring.

## Introduction

IoT enabled Wireless Sensor Network (WSN) monitoring infrastructure is a sustainable, eco-friendly, and economical way of data collection approach that enable high quality and self-sustainable crop production with optimum utilization of resources^1,2^. Sensing coverage and connectivity optimization is a fundamental design problem in WSN and is an implication of the initial Node Deployment Strategy (NDS)^3^. The K-Coverage strategy, where each location is at least within the *k* node communication range, provides a measure of WSN deployment Quality of Service (QoS). Increasing the coverage of WSNs increases the success rate in performing specific sensing operations. The selection of *k* comes down to a trade-off between coverage and node-count. The two factors have a negative correlation, and their choice impacts the overall effectiveness of WSN deployment^4^. The coverage is also closely related to network connectivity. In the literature, proposals are made to realize K-connectivity $\left( k\ge 1 \right)$. This means that there are at least *k* disjoint paths between a pair of sensors^5^. Connectivity is critical to ensure that the data acquired by the sensor can be routed to the Base-station. Overall, an NDS influences the coverage, connectivity, and cost of a WSN deployment. In a deterministic NDS, nodes are placed with careful planning of separation distances, elevations, and node orientations, to achieve a deployment where all nodes fall within each other’s communication range^6^. The NDS in arable land before sowing should envisage crop height and density at the maturity stage to estimate potential signal attenuation, which has been ignored in recent developments^7–10^. In the literature, NDSs assume that nodes are in a direct line-of-sight, overlooking the fact that when deployed for crop monitoring, the network cannot withstand increased signal attenuation as vegetation increases. The $2.4\;{\text{GHz}}$ Radio Frequency has theoretically higher propagation losses, which makes radio coverage management more challenging compared to 868 and $920\;{\text{MHz}}$ low-frequency bands applied by WSN; however, it can provide higher data transmission. For that reason, when the approaches by Wu et al.^11^ and, Guo and Jafarkhani^12^ were implemented to monitor the MP-3713 wheat crop using the IEEE 802.15.4 communication standard, the network faced dis-connectivity due to increased signal attenuation in the stages of grain-filling and maturity. IoT-based agricultural farm monitoring infrastructure has been proposed in by Ramli et al.^13^, Heble et al.^14^, Yim et al.^15^, Davcev et al.^16^ and Farooq et al.^17^. Ongoing studies have investigated the radio propagation in the forest environment^18,19^. The In-depth radio propagation investigations such as the small-scale fading and shadowing loss of the narrowband channel and the characteristics of the ultra-wideband (UWB) channel were modeled empirically^20,21^. These empirical models in the forest environment provide beneficial information for radio propagation in agricultural areas^22^. Specific parameters of the developed propagation channel can be applied to orchards due to similarity in trunk pattern. However, their implementation in the food grass environment can be challenging. For Instance, the authors in Dhanavanthan et al.^23^ empirically fitted the measurement results for a corn field at 2.4 GHz by using the model’s parameters recommended for the forest scenario. They reported depreciation in estimated path loss over measured value, especially during the crop maturity stage. Recently, measurements have been made at different frequencies and antenna heights in agricultural fields^18,19^. For example, in Ndzi et al.^24^, the authors compare the path loss in the 2.45 GHz band at antennas height 0.15 m and 1 m in cashew, cornfield and herb field. They concluded that the path loss difference in scenarios with $0.15\;{\text{m}}$ antenna height in 10 m of vegetation depth is $\approx 37$ higher than in scenarios with $1\;{\text{m}}$ antenna. They claimed that the difference in path loss between the two antennas in herb is large $( \approx 20\;{\text{dB}})$, due to the fact that the height of the herbs being less than $1\;{\text{m}}$. However, none of these approaches discuss the effect of vegetation height and density on $NDS^{z}$.

The article "Genetic algorithm optimized node deployment in IEEE 802.15.4 potato and wheat crop monitoring infrastructure" was published in 2021. Journal: Sci Rep.

In Bayrakdar et al.^25^ authors, minimize node deployment in agricultural farms through the deterministic placement of nodes using a node separation aware fuzzy logic approach. In Soman et al.^26^, A Genetic Algorithm (GA)-based optimization strategy was proposed to identify the minimum number of nodes to implement a Guided Wave-Based Damage Detection system for structural health monitoring. In a similar GA based approach in ZainEldin et al.^27^, authors maximized the area coverage with the lowest number of nodes and minimized overlapping areas between neighboring nodes. In Phoemphon et al.^28^, the authors proposed a particle swarm optimization (NS-IPSO) node segmentation approach that divides nodes into segments to improve the accuracy of the estimated distances between pairs of anchor nodes and unknown nodes. All these implementations consider the application scenario as a static environment, and the effect of changing density due to increasing vegetation height on RSSI has been overlooked. Compared to the work presented in the literature, the NSGA-II based node placement optimization in this work ensures the convergence toward global optimum solutions. The NSGA-II is widely used in many application scenarios due to the diversity in solutions, and ideal convergence to the Pareto optimum solutions^29^. The NSGA-II has several reference points, which usually are widely distributed in standardized hyperplanes to maintain diversity. For these reference points, the algorithm can find a solution close to the Pareto optimal. This work’s novelty is two-fold, first, capturing the effect of increasing vegetation density on RSSI of IEEE 802.15.4 WSN infrastructure through path loss coefficient formulation of log-normal path loss shadowing model. Second, RSS based NSGA-II optimized node deployment strategy.

In this work, we have developed an IEEE 802.15.4 based real-time monitoring infrastructure in potato and wheat crops to capture the effect of vegetative growth on Received Signal Strength (RSS) and network connectivity. Further, we have employed the derived RSS measurements to optimize NDS in wheat (MP-3173) and potato (Kufri Jawahar) crop over coverage, connectivity, and cost using NSGA-II multi-objective evolutionary computation. Contributions of the proposal are as follow:

- Design and deployment of a real-time IEEE 802.15.4 standard WSN crop monitoring infrastructure for RSS analysis in wheat (MP-3173) and potato (Kufri Jawahar) crop.
- Identification of the path loss coefficient $\eta$ for $2.4\;{\text{GHz}}$ radio signal in different growing stages of target crops.
- Design of RSS based NSGA-II optimized Node Deployment Strategy (NSGAII-NDS).

The article "Genetic algorithm optimized node deployment in IEEE 802.15.4 potato and wheat crop monitoring infrastructure" was published in 2021. Journal: Sci Rep.

The paper is organized as follow. Section 2 presents the problem formulation and related work. In Section 3, the proposed NSGA-II optimized node deployment strategy is presented. Section 4, validate the effectiveness of proposed approach and finally, in Section 5, conclusions are drawn.

## Problem definition

This section presents real-time WSN deployment setup details in wheat and potato crops, i.e., Experiment-1 and Experiment-2. Further, the problem has been analyzed to develop an effective NDS by discussing experimental observations.

### Experimentation setup

The number of sensor nodes |*N*|, in Experimentation-1 and Experimentation-2 are, $\left| N^{wheat} \right| =25$ and $\left| N^{potato} \right| =10$, i.e., $N^{potato}=\left\{ n_{1}^{potato},n_{1}^{potato},\cdots ,n_{i}^{potato},\cdots , n_{10}^{potato} \right\}$ and $N^{wheat}= \{ n_{1}^{wheat},n_{1}^{wheat},\cdots ,n_{i}^{wheat},\cdots , n_{25}^{wheat} \}$. Nodes in the network are running the Contiki-ng operating system that implements the $\mu ip6$ communication stack and use the IEEE-802.15.4 supported ContikiMAC link layer protocol for radio duty cycle power consumption management. The main controller and gateway in Sink node are designed using Raspberry-pi and CC2530 packet sniffer. The target areas are part of Maharajpura Farmland, Gwalior, Madhya-Pradesh, India^30^. The position of $n_i^x$ in target area $T^x \mid x \in \{wheat,potato\}$ of dimension $( D^{T^{^{x}}}_{L} \times D^{T^{^{x}}}_{B})$ meters, are the latitude and longitude coordinate values $(n_{i^{^{lat}}}^{x},n_{i^{^{lon}}}^{x})$ . For tractability, $T^x$ is visualised as a grid of size $(1 \times 1)m$ square cells. Thus, $T^x$ is modeled as a lattice $H^{x}\left[ {\overline{D}}^{T^{^{x}}}_{L} \right] \left[ {\overline{D}}^{T^{^{x}}}_{B} \right] \bigl \vert {\overline{D}}^{T^{^{x}}}_{L}=\left\lceil \frac{D^{T^{^{x}}}_{L}}{d} \right\rceil , {\overline{D}}^{T^{^{x}}}_{B}=\left\lceil \frac{D^{T^{^{x}}}_{B}}{d} \right\rceil$ . After discretisation, sensor node $n_i^x$ situated at $(n_{i^{^{lat}}}^{x},n_{i^{^{lon}}}^{x})$ is in the cell $H^{x}\left[ y \right] \left[ z \right]$, where *y* and *z* are calculated as follow:

1 $$\begin{aligned} y=\left\lceil \frac{\left| {\overline{n}}_{i^{^{lat}}}^{x} -n_{i^{^{lat}}}^{x} \right| }{d} \right\rceil , z= \left\lceil \frac{\left| {\overline{n}}_{i^{^{lon}}}^{x} -n_{i^{^{lon}}}^{x} \right| }{d} \right\rceil \end{aligned}$$

Here $({\overline{n}}_{i^{^{lat}}}^{x},{\overline{n}}_{i^{^{lon}}}^{x})$ is the location of node positioned in the first cell, i.e. $H^{x}[0][0]$. To model coverage and over-coverage issue, a counter $C^{x}\left[ y \right] \left[ z \right]$ is assigned to each cell $H^{x}\left[ y \right] \left[ z \right]$ in $T^x$, representing the number of time a point covered by underlying sensor infrastructure. The outcome of this counter implementation will be a counter map of dimension $C^{x} [ {\overline{D}}^{T^{^{x}}}_{L} ] [ {\overline{D}}^{T^{^{x}}}_{B} ]$, where each counter value $C^{x}\left[ y \right] \left[ z \right]$ is associated to a grid cell $H^{x}\left[ y \right] \left[ z \right]$. Initially $C^{x}\left[ y \right] \left[ z \right]$ is set to 0 and is incremented if $H^{x}\left[ y \right] \left[ z \right]$ is in the communication range of $n_i^x$. For example, if $H^{x}\left[ y_1 \right] \left[ z_1 \right]$ and $H^{x}\left[ y_2 \right] \left[ z_2 \right]$ are in the communication range of two and three sensor nodes, then respective counter values will be $C^{x}\left[ y_1 \right] \left[ z_1 \right] =2$ and $C^{x}\left[ y_2 \right] \left[ z_2 \right] =3$. In experimentation-1 target farmland $T^{wheat}$ has composite symmetry $(lat-26.312131 ^{\circ }, lon-78.220099 ^{\circ })$, with an area of $\approx 8.04 \times 10^{4} \;{\text{m}}^{2}$. The period of observation started from $23 \ November \ 2019$ with the sowing of MP-3173 Wheat, and ended on $4 \ March \ 2020$. In experimentation-2 Target farmland $T^{potato}$ has rectangular symmetry $(lat-26.313247 ^{\circ }, lon-78.223374 ^{\circ })$, with an area of $\approx 7.53 \times 10^{4} \;{\text{m}}^{2}$. The period of observation started on $28 \ June \ 2019$, with sowing of kufri-jawahar potato and ended on $30 \ October \ 2019$. The soil composition, and adopted potato and wheat plantation strategy is presented in reports by Panigrahi et al.^31^ and Devi et al.^32^, respectively.

The article "Genetic algorithm optimized node deployment in IEEE 802.15.4 potato and wheat crop monitoring infrastructure" was published in 2021. Journal: Sci Rep.

**Figure 1:** Sensor node prototype and deployment in $T^{wheat}$ and $T^{potato}$.

### Sensor architecture

The devised sensor node $n_i$ prototype is shown in Fig. 1. The $n_i$ control-unit is designed using *CC*2538 wireless Microcontroller System-On-Chip for 2.4-GHz IEEE 802.15.4 and is powered by two parallel-connected Panasonic $CR1632-3V$ lithium coin cells^33^. The *CC*2538 transceiver output power, which has a receiving sensitivity $- 97\;{\text{dBm}}$ in low-gain mode, is programmed to $7\;{\text{dBm}}$ and is connected to a $3\;{\text{dB}}$ gain planer inverted $\ F$-antenna^34^. The alignment of the XY-plane of the antenna in deployed $n_{i}^{x}$ is orthogonal to the XY-plane of $T^{x}\mid x \in \{ wheat,potato \}$. A node is equipped with a resistive soil moisture sensor, photoresistor, and TMP36 temperature sensor. To protect the nodes from environmental hazards, they are enclosed in a PVC enclosure and installed on top of a hollow aluminum tube, which, upon deployment in $T^{x}$, gives the $n_{i}^{x}$ antenna an elevation of $32\;{\text{cm}}$ from ground.

### Path-loss model and RSSI evaluation

The *CC*2538 has built-in RSSI functionality, which calculates an 8-bit signed digital value and can be automatically read from the received frame or incoming packet. The RSS value captured by RSSI is a 2s-complement signed number on a logarithmic scale with 1-dB steps. An offset is added to RSSI value to find actual signal power *P* accurately, i.e, $P= RSSI-offset (dB)$. The RSSI offset value in contiki for *CC*2538 is set to $73\ dB$. The measured RSSI readings for wheat crop in sowing and flowering stages are shown in Fig. 2. The Discrete Cosine Transform (DCT) interpolation technique has been used to develop the RF map from the RSS-sample dataset^35^. The employed path-loss model is the Log-Normal Shadowing and is represented by Eq. 2.

2 $$\begin{aligned} PL\left( d_{\left( n_i,n_j \right) } \right)= & {} PL\left( d_{\left( n_i,n_o \right) } \right) + 10\eta \log _{10}\left( \frac{d_{\left( n_i,n_j \right) }}{d_{\left( n_i,n_o \right) }} \right) + {{\chi }}_{\sigma } \end{aligned}$$

3 $$\begin{aligned} PL\left( d_{\left( n_i,n_o \right) } \right)= & {} -10 \log \left( \frac{P_{n_i}^{t}}{P_{n_o}^{r}} \right) =-10 \log \left( \frac{G_{n_i}^{t}G_{n_o}^{r}\lambda ^2}{\left( 4 \pi d_{\left( n_i,n_o \right) } \right) ^2} \right) \end{aligned}$$

where $PL\left( d_{\left( n_i,n_o \right) } \right)$ is the reference path loss between node $n_i$ and $n_o$ at distance $d_{\left( n_i,n_o \right) }$ , $\eta$ is the path loss exponent and $\chi _{\sigma }$ is a Gaussian distributed random variable with zero mean and $\sigma$ standard deviation. For the calculation of $\eta$, the collected empirical measurements of RSS are analyzed using Eq. 4.

4 $$\begin{aligned} f\left( \eta \right)= & {} \sum _{l=1}^{k}\left( P^{rec} \big (d_{\left( n^{ref},n_i \right) }^l \big )-P^{est} \big (d_{\left( n^{ref},n_i \right) }^l \big ) \right) ^2 \nonumber \\= & {} \sum _{l=1}^{k} \Bigg ( P^{rec} \big (d_{\left( n^{ref},n_i \right) }^l \big ) - {\overline{P}}^{est} \left( d_{\left( n^{ref},n_o \right) }^l \right) +10 \log {\frac{d_{\left( n^{ref},n_i \right) }^l}{d_{\left( n^{ref},n_o \right) }^l}} \Bigg )^2 \end{aligned}$$

where $P^{rec} \big (d_{\left( n^{ref},n_i \right) }^l \big )$ is the received power and $P^{est} \big (d_{\left( n^{ref},n_i \right) }^l \big )$ is the estimated power at distance $d^l$. The value of $\eta$ is identified by minimizing the mean square error between $P^{rec} \big (d_{\left( n^{ref},n_i \right) }^l \big )$ and $P^{est} \big (d_{\left( n^{ref},n_i \right) }^l \big )$ presented in Eq. 4. The RSS samples are taken from database acquired through continuous and periodic measurements. Continuous measurements were collected using sensor nodes deployed in Experiments 1 and 2 with a 30 minutes sampling rate. The periodic measurements were collected at intervals of 4 days using the HSA2030 Spectrum analyzer, operating in zero-span mode. The data sets are classified based on the distance $d_{\left( n_i,n^{ref} \right) }$ from a reference node $n^{ref}$ in different growing stages of the target crop. The selected $n^{ref}$ is placed at the nucleus of $T^x \mid \left\{ wheat,potato \right\}$, and the remaining $n_i^x$ is positioned around $n^{ref}$ using approach by Wu et al.^11^. To obtain $\eta$, the RSS data is analyzed by evaluating a total of 1500 and 1600 samples in Eq. 4. The $\eta$ calculated for two crops in different growing stages is presented in Table 1. The range $P_{lim}^{r} \left( {\overline{d}}_{\left( n_i,n_j \right) } \right)$ attained by *CC*2538 sensor node with $- 97\;{\text{dBm}}$ sensitivity in the free space environment, after incorporating the losses incurred by the enclosure, is measured to be $\approx 63\;{\text{m}}$. The Outage probability $Prob\left( P^r \left( d_{\left( n_i,n_j \right) } \right) < P_{lim}^{r} \left( {\overline{d}}_{\left( n_i,n_j \right) } \right) \right)$ of $93\%$ at $- 75\;{\text{dBm}}$ with margin ${\overline{P}}^r \left ( d_{\left( n_i,n_j \right) } \right )- P_{lim}^{r} \left( {\overline{d}}_{\left( n_i,n_j \right) } \right)$ of $8\;{\text{dBm}}$ is employed and is identified using formulation presented in Eq. 5.

5 $$\begin{aligned} Prob{\text{ }}\left( {P^{r} \left( {d_{{\left( {n_{i} ,n_{j} } \right)}} } \right) < P_{{lim}}^{r} \left( {\bar{d}_{{\left( {n_{i} ,n_{j} } \right)}} } \right)} \right) & = \frac{1}{{\sqrt {2\pi } \sigma }}\int_{\beta }^{\infty } {e^{{\frac{{ - x^{2} }}{{2\sigma ^{2} }}}} } \;dx = Prob\left[ {\bar{P}^{r} d_{{\left( {n_{i} ,n_{j} } \right)}} - \chi _{\sigma } < P_{{lim}}^{r} \left( {\bar{d}_{{\left( {n_{i} ,n_{j} } \right)}} } \right)} \right] \\ & \quad = Q\left( {\frac{{\bar{P}^{r} d_{{\left( {n_{i} ,n_{j} } \right)}} - P_{{lim}}^{r} \left( {\bar{d}_{{\left( {n_{i} ,n_{j} } \right)}} } \right)}}{\sigma }} \right) = \frac{1}{2}\left( {\frac{{\bar{P}^{r} d_{{\left( {n_{i} ,n_{j} } \right)}} - P_{{lim}}^{r} \left( {\bar{d}_{{\left( {n_{i} ,n_{j} } \right)}} } \right)}}{{\sqrt 2 \sigma }}} \right) \\ \end{aligned}$$

**Figure 2:** Latitude,longitude representation and RSS measurement in $T^{wheat}$. MATLAB 2016a. https://in.mathworks.com/.

The article "Genetic algorithm optimized node deployment in IEEE 802.15.4 potato and wheat crop monitoring infrastructure" was published in 2021. Journal: Sci Rep.

With a sensitivity of $- 75\;{\text{dBm}}$ in the free-space environment, the measured transmission range of node $n_i$ is identified to be $\approx 48\;{\text{m}}$.

**Table 1:** The calculated $\eta$ for two crops in different growing stages.

Potato				Wheat			
Stage	Period	Days	$\varvec{\eta }$	Stage	Period	Days	$\varvec{\eta }$
Establishment	28/06/2019–20/07/2019	23	1.83	Floral Initiation	24/11/2019–13/12/2019	19	1.85
Stolon Initiation	21/07/2019–09/08/2019	20	2.47	T–Spikelet Initiation	14/12/2019–07/01/2020	24	2.75
Tuber Initiation	10/08/2019–29/08/2019	19	2.71	Heading	08/01/2020–28/01/2020	20	3.94
Tuber filling	30/08/2019–12/10/2019	43	2.83	Grain FillingPeriod	29/01/2020–28/02/2020	30	6.21
Maturity	13/10/2019–29/10/2019	16	2.76	physiological Maturity	29/02/2020–20/03/2020	20	5.93

*Software tool*: The prepossessing of collected RSSI measurement is done using Hadoop and Spark environment. The environment is setup on an Intel Xeon Processor E5 Family workstation which is running an Ubantu 18.4 operating system. The path loss model is implemented using Python programming language and the results are generated using MATLAB numeric computing environment.

### Experiment observations

In both the experiments, nodes were deployed before the crop sowing stages using the strategy presented by Wang et al.^36^. The key observation in Experiment-2 over wheat crop was the reduced RSSI measurement over time, eventually leading to link drop and network dis-connectivity. This phenomenon has been observed to occur in three stages of wheat growth, namely terminal-spikelet initiation, heading, and physiological maturity. The network dis-connectivity caused by link drop was due to an increase in signal attenuation from growth in vegetation density. Since the initial deployment was done on the fact that $\eta = 1.85$, the receiving sensitivity of $- 75\;{\text{dBm}}$ between $n_i$ and $n_j$ was estimated to be at a distance of $\approx 48\;{\text{m}}$. However, factors such as vegetation height, density, and plating strategy have affected $\eta$. When measured using Eq. 4 in maturity stage, it is found to be $\eta =5.93$, which is $\approx 8\;{\text{m}}$ at $- 75\;{\text{dBm}}$ receiving sensitivity for uninterrupted link communication. On the contrary, the RSSI measurement for potato crop through out the season was consistent.The measured $\eta$ in the sowing and maturity stage was found to be, 1.83 and 2.76. The Kufri Jawahar potato plant, which can attain elevation up to $34\;{\text{cm}}$ at maturity, has little effect on the transmitted signal of $n_{i}^{wheat}$, as it is located at the height of $32\;{\text{cm}}$ from the ground and is out of the vegetation canopy.

The article "Genetic algorithm optimized node deployment in IEEE 802.15.4 potato and wheat crop monitoring infrastructure" was published in 2021. Journal: Sci Rep.

*Summary*: Two conclusions were drawn based on the observation made in Experiment 1 and 2 and are as follows:

- An NDS developed for crop *X* with $\eta ^x$, if used in crop *Y* with $\eta ^y$, may cause network over-coverage in the case of $\eta ^{x}<\eta ^{y}$ and network dis-connectivity if $\eta ^{x}>\eta ^{y}$.
- The path loss coefficient $\eta ^z$ in target crop $T^z$ should be identified before the $NDS^{z}$ formulation.

In addition to the work done in Ndzi et al.^24^, Ding *et al.*^18^ and Olasupo et al.^19^ we have collected RSS samples for a crop cycle in a multi-hop communication scenario for better path loss modeling in potato and wheat crop. Next to this, we have developed an optimal node placement strategy to deploy a practical real-time crop monitoring infrastructure by integrating derived PLC to NSGAII-NDS.

## NSGA-II based NDS optimization (NSGAII-NDS)

In this section, a multi-objective crop dependent node deployment strategy $NDS^{z}$ is proposed. The flow-chart of proposed model is presented in Fig. 3. The outcome is a set of $\left( n_{i^{lat}}^{x},n_{i^{lon}}^{x} \right) \mid n_{i}^{x} \in N^x, x \in \left\{ wheat,potato \right\}$, optimized using elitist Non-dominated Sorting Genetic Algorithm (NSGA-II) on coverage, over-coverage, and RSS. The NSGA-II is widely used in many application scenarios due to diversity in solution and more desired convergence near the true Pareto optimal set^37^.

**Figure 3:** Proposed NSGA-II optimized node deployment strategy flow-diagram.

### Chromosome representation

Genetic Algorithm (GA)based optimization is comprised of chromosome $Chr^{x}$ representing a possible solution $NDS^{z}$ and Population $Pou^{T^x}$, which is a collection of these chromosomes. The $Chr^{x}$ in GA is derived from the phenotype, a single design factor composed of a domain of values. In the given scenario, node’s latitude and longitude value $\left( n_{i^{lat}}^{x},n_{i^{lon}}^{x} \right)$ and transmission range ${{\mathscr {T}}}^{N^{x}}$ are Phenotype design factors that are mapped to Genotype using Real value Encoding with Binary Codes (REBC). The phenotype-genotype relationship for $NDS^{wheat}$ is shown in Table 2. Genomes in a binary string form are converted to real value using the REBC reverse mapping rule. The *REBC* mapping schema transforms a continuous real-valued PHEnotype (PHE) design variable ${{\mathscr {X}}}_{i}^{PHE} \mid {{{\mathscr {X}}}}_{min}^{PHE}\le {{{\mathscr {X}}}}_{i}^{PHE} \le {{{\mathscr {X}}}}_{max}^{PHE}$ into a binary string of length $\overline{{{\mathscr {B}}}}_{i}^{PHE} \mid \overline{{{\mathscr {B}}}}_{i}^{PHE}=\left\lceil {{{\mathscr {B}}}}_{i}^{PHE} \right\rceil$ and is derived as follows:

6 $$\begin{aligned} \overline{{{\mathscr {B}}}}_{i}^{PHE}=\left\lceil {{{\mathscr {B}}}}_{i}^{PHE} \right\rceil =\left\lceil \log _{2}\left( \frac{\overline{{{\mathscr {X}}}}_{max}^{PHE}- \overline{{{\mathscr {X}}}}_{min}^{PHE}}{{{\mathscr {E}}}} \right) \right\rceil \end{aligned}$$

where ${{\mathscr {E}}}$ is conversion precision factor, i.e., if ${{\mathscr {E}}}=0.02$ then $4.02=3.98=4$. For $NDS^{potato}$, we have a total of eleven design factors, 10 for $n_{i}^{potato} \mid n_{i}^{potato} \in N^{potato}, \left| N^{potato} \right| =10$, and one for ${{\mathscr {T}}}^{potato}$. For $NDS^{wheat}$, we have a total of 26 design factors, 25 for $n_{i}^{wheat} \mid n_{i}^{wheat} \in N^{wheat}, \left| N^{wheat} \right| =25$, and one for ${{\mathscr {T}}}^{wheat}$, Table 2. The binary equivalent of real value is the binary representation of $\overline{{{\mathscr {X}}}}_{i}^{PHE}$ and is derived as follows:

7 $$\begin{aligned} {{{\mathscr {X}}}}_{i}^{PHE}= {{{\mathscr {X}}}}_{min}^{PHE}+\frac{ {{{\mathscr {X}}}}_{max}^{PHE}- {{{\mathscr {X}}}}_{min}^{PHE}}{2^{n}-1} \times \overline{{{\mathscr {X}}}}_{i}^{PHE} \overline{{{\mathscr {X}}}}_{i}^{PHE}= \frac{\left( {{{\mathscr {X}}}}_{i}^{PHE} - {{{\mathscr {X}}}}_{min}^{PHE} \right) \left( {2^{n}-1}\right) }{{{{\mathscr {X}}}}_{max}^{PHE}- {{{\mathscr {X}}}}_{min}^{PHE}} \end{aligned}$$

The range of ${{\mathscr {T}}}^{x}$ and $\left( n_{i^{lat}}^{x},n_{i^{lon}}^{x} \right)$ design variables, $\left[ {{{\mathscr {X}}}}_{min}^{PHE}, {{{\mathscr {X}}}}_{max}^{PHE} \right] \mid {{{\mathscr {X}}}}_{min}^{PHE}< {{{\mathscr {X}}}}_{max}^{PHE}$, is derived from Table 2. The initial values of the design variables are randomly generated within the predefined range and then optimized over coverage, over-coverage and RSS in sorting, mutation and crossover phases of the NSGA-II.

The article "Genetic algorithm optimized node deployment in IEEE 802.15.4 potato and wheat crop monitoring infrastructure" was published in 2021. Journal: Sci Rep.

**Table 2:** The range of ${{\mathscr {T}}}^{x}$ and $\left( n_{i^{lat}}^{x},n_{i^{lon}}^{x} \right)$ design variables and Phenotype-Genotype representation.

Design variable	$n_{i^{lat}}^{potato}$	$n_{i^{lon}}^{potato}$	${{\mathscr {T}}}^{potato}$	$n_{i^{lat}}^{wheat}$				$n_{i^{lat}}^{wheat}$				${{\mathscr {T}}}^{wheat}$
VariableMaximum ${{{\mathscr {X}}}}_{min}^{PHE}$	$26.280432 ^{\circ }$	$26.280432 ^{\circ }$	$-99 \ dBm$	$26.280432 ^{\circ }$	$26.280432 ^{\circ }$	$26.280432 ^{\circ }$	$26.280432 ^{\circ }$	$26.280432 ^{\circ }$	$26.280432 ^{\circ }$	$26.280432 ^{\circ }$	$26.280432 ^{\circ }$	$-99 \ dBm$
Minimum ${{{\mathscr {X}}}}_{max}^{PHE}$	$26.280432 ^{\circ }$	$26.280432 ^{\circ }$	$-99 \ dBm$	$26.280432 ^{\circ }$	$26.280432 ^{\circ }$	$26.280432 ^{\circ }$	$26.280432 ^{\circ }$	$26.280432 ^{\circ }$	$26.280432 ^{\circ }$	$26.280432 ^{\circ }$	$26.280432 ^{\circ }$	$-99 \ dBm$
	** PHENOTYPE**											

	$n_{1}^{wheat}$		$n_{2}^{wheat}$		$n_{3}^{wheat}$		$n_{4}^{wheat}$		$\cdots$	$\cdots$	$n_{25}^{wheat}$	
	$n_{1^{lat}}^{wheat}$	$n_{1^{lon}}^{wheat}$	$n_{2^{lat}}^{wheat}$	$n_{2^{lon}}^{wheat}$	$n_{3^{lat}}^{wheat}$	$n_{3^{lon}}^{wheat}$	$n_{4^{lat}}^{wheat}$	$n_{4^{lon}}^{wheat}$	$\cdots$	$\cdots$	$n_{25^{lat}}^{wheat}$	$n_{25^{lon}}^{wheat}$
	26.281885r̆	78.223802r̆	26.281007r̆	78.223072r̆	26.281872r̆	78.223532r̆	26.281117r̆	78.223192r̆	$\cdots$	$\cdots$	26.280124r̆	78.220254r̆
${{\mathscr {B}}}_{i^{(lat,lon)}}^{wheat}$	184	224	166	209	157	183	201	215	$\cdots$	$\cdots$	147	151
$\overline{{{\mathscr {B}}}}^{total}$	8	8	8	8	8	8	8	8	$\cdots$	$\cdots$	8	8
Index	[0-7]	[8-15]	[16-23]	[24-31]	[32-39]	[40-47]	[48-55]	[56-63]	$\cdots$	$\cdots$	[384-391]	[392-399]
$Chr_{{{\mathscr {X}}}}[i]$	10111000	11100000	10100110	11010001	10011101	10110111	11001001	11010111	$\cdots$	$\cdots$	10010011	10010111
	** GENOTYPE**											

### Multi-objective functions 

The non-dominated sorting to obtain $NDS^{z}$ arranges the chromosome $chr^{x}[i]$ in each generation based on the fitness toward objectives $\overline{{{\mathscr {O}}}}^{total}=\left\{ {{\mathscr {O}}}^{Cov},{{\mathscr {O}}}^{Ocov},{{\mathscr {O}}}^{RSS} \right\}$. The $NDS^{z}$ befitting requires maximum coverage ${{\mathscr {O}}}^{Cov}$, minimum over-coverage ${{\mathscr {O}}}^{Ocov}$ and improved signal strength ${{\mathscr {O}}}^{RSS}$. The goal of ${{\mathscr {O}}}^{Cov}$ in Eq. 8 is to maximize agricultural farm $T^x$ coverage, that is, to increase the count of grid cell $H^{x}\left[ y \right] \left[ z \right]$ in the communication of deployed sensor nodes $N^x$, i.e. $\forall C^{x}\left[ y \right] \left[ z \right] \ne 0$ .

8 $$\begin{aligned}&{{\mathscr {O}}}^{Cov} \left( chr^{x}[i] \right) = \max \limits _{i \in {{\mathscr {I}}}} \left( Cov\left( chr^{x}[i] \right) \right) = \max \limits _{i \in {{\mathscr {I}}}} \left\{ \sum _{i=0}^{\left( {\overline{D}}_{L}^{T_x} -1\right) } \sum _{j=0}^{\left( {\overline{D}}_{B}^{T_x} -1\right) } C_{Cov}^{x}[i][j]\right\} , \nonumber \\&C_{Cov}^{x}[i][j]=\left\{ \begin{matrix}1 &{} if \ \ C^{x}[i][j] \ne 0\\ 0 &{} otherwise \end{matrix}\right. \end{aligned}$$

The second objective ${{\mathscr {O}}}^{Ocov}$ presented in Eq. 9 aims to minimize over-coverage by reducing the count of those grid cells $H^{x}\left[ y \right] \left[ z \right]$ which are in the communication range of more than *k* sensor nodes, i.e. $\forall C^{x}\left[ y \right] \left[ z \right] > 3$.

9 $$\begin{aligned}&{{\mathscr {O}}}^{Ocov} \left( chr^{x}[i] \right) = \min \limits _{i \in {{\mathscr {I}}}} \left( Ocov\left( chr^{x}[i] \right) \right) = \min \limits _{i \in {{\mathscr {I}}}} \left\{ \sum _{i=0}^{\left( {\overline{D}}_{L}^{T_x} -1\right) } \sum _{j=0}^{\left( {\overline{D}}_{B}^{T_x} -1\right) } C_{Ocov}^{x}[i][j]\right\} , \nonumber \\&C_{Ocov}^{x}[i][j]=\left\{ \begin{matrix} C^{x}[i][j] &{} if \ \ C^{x}[i][j]>3\\ 0 &{} otherwise \end{matrix}\right. \end{aligned}$$

Third objective ${{\mathscr {O}}}^{RSS}$, Eq. 10, aims to increase the received signal strength between two sensor nodes. The ${{\mathscr {O}}}^{RSS}$ ensures the connectivity by  identifying the distance at which the RSSI remain consistent throughout the lifetime of network. The $PL\left( d_{\left( n_i,n_j \right) } \right)$ is the path loss between node $n_i^x$ and $n_j^x$, and is formulated in Eq. 2.

10 $$\begin{aligned} {{\mathscr {O}}}^{RSS} \left( chr^{x}[i] \right) = \max \limits _{i \in {{\mathscr {I}}}} \left( RSS\left( chr^{x}[i] \right) \right) = \max \limits _{i \in {{\mathscr {I}}}} \left\{ \sum _{i=1}^{\left| N^x \right| } \sum _{j=1}^{\left| N^x \right| } PL\left( d_{\left( n_i,n_j \right) } \right) \right\} \end{aligned}$$

The article "Genetic algorithm optimized node deployment in IEEE 802.15.4 potato and wheat crop monitoring infrastructure" was published in 2021. Journal: Sci Rep.

### Initial population generation

The Initial Population Generation (IPG) initiates the NSGA-II operation by seeding a set of possible solutions from a universe of solutions in between the lower and upper bound of the design variables. The minimum and maximum range of design variables required for IPG operations were identified and are presented in Table 2. In order to avoid premature convergence, the diversity in IPG needs to be maintained, and this has been achieved by the heuristic initialization of the population, followed by a probabilistic distribution. The approach’s fundamental design components, i.e., search space, number of individuals, problem difficulty and fitness functions, and influencing solution diversity, have been taken into account during the IPG process. The former seeding approach avoids premature convergence of ${{\mathscr {T}}}^{N^{x}}$ and $\left( n_{i^{lat}}^{x},n_{i^{lon}}^{x} \right)$ optimization. The population’s diversity has been evaluated at three levels, i.e., gene level, chromosome level, and population level. The gene-level diversity formulation in Eq. 11 is a bias measure ${{\mathscr {P}}}_{t}^{bias}$ presented by Diaz-Gomez *et al.*^38^. Where $\overline{{{\mathscr {B}}}}_{i}^{total}$ is the length of a chromosome $chr^{x}$, ${{\mathscr {I}}}_t$ is the total number of $chr^{x}$, and $chr^{x} \left[ i \right] \left[ j \right]$ is the $j$th gene of $i$th chromosome. The elements of ${{\mathscr {P}}}_{t}^{bias}$ are distributed over the range $\left[ 0.5, 1.0 \right]$, where the value closer to 0.5 is comparatively more stable.

11 $$\begin{aligned} {{\mathscr {P}}}_{t}^{bias}=\frac{1}{\overline{{{\mathscr {B}}}}_{t}^{total} \times {{\mathscr {I}}}_t}\sum _{j=1}^{\overline{{{\mathscr {B}}}}_{t}^{total}} \max \left\{ \sum _{i=1}^{{{\mathscr {I}}}_t}\left( 1-chr^{x}\left[ i \right] \left[ j \right] \right) ,\sum _{i=1}^{{{\mathscr {I}}}_t} chr^{x}\left[ i \right] \left[ j \right] \right\} \end{aligned}$$

Chromosome-level diversity in Eq. 12 is the average Hamming distance ${{\mathscr {P}}}_{t}^{HD}$ among the $chr^{x}$ in the population. Two chromosomes $chr^{x}{[i]}$ and $chr^{x}{[j]}$ are distinct if their ${{\mathscr {P}}}_{t}^{HD}$ is equal to $chr^{x}$ length, i.e., ${{\mathscr {P}}}_{t}^{HD}=\overline{{{\mathscr {B}}}}_{i}^{total}$.

12 $$\begin{aligned} \overline{{{\mathscr {P}}}}_t^{HD}= & {} 2 \times \sum _{i=1}^{{{\mathscr {I}}}_t} \sum _{j=i+1}^{{{\mathscr {I}}}_t} {{\mathscr {P}}}_t^{HD}\left( chr^{x}\left[ i \right] , chr^{x}\left[ j \right] \right) \nonumber \\= & {} 2 \times \sum _{i=1}^{{{\mathscr {I}}}_t} \sum _{j=i+1}^{{{\mathscr {I}}}_t} \left( \sum _{n=1}^{\overline{{{\mathscr {B}}}}_t^{total}}\left( \left| chr^{x}\left[ i \right] \left[ n \right] - chr^{x}\left[ j \right] \left[ n \right] \right| \right) \right) \end{aligned}$$

Population-level diversity, determined by Eq. 13, identifies the Centre of Mass (CoM) of the population matrix, here $chr^{x} \left[ 0 \right] \left[ 0 \right]$ and $chr^{x} \left[ {{\mathscr {I}}}_t \right] \left[ \overline{{{\mathscr {B}}}}_{i}^{total} \right]$ are the first and last indexes of the matrix. The $CoM_1^x$ gives the CoM of an *x* coordinate with value 1, and equation $CoM_1^y$ identifies the CoM of *y* coordinate with value 1.

13 $$\begin{aligned} CoM_1^x=\frac{\sum _{i=1}^{{{\mathscr {I}}}_t}\sum _{j=1}^{\overline{{{\mathscr {B}}}}_t^{total}}col \left( chr^{x} \left[ i \right] \left[ j \right] \right) }{\sum _{i=1}^{{{\mathscr {I}}}_t}\sum _{j=1}^{\overline{{{\mathscr {B}}}}_t^{total}} chr^{x} \left[ i \right] \left[ j \right] },CoM_1^y=\frac{\sum _{i=1}^{{{\mathscr {I}}}_t}\sum _{j=1}^{\overline{{{\mathscr {B}}}}_t^{total}} row \left( chr^{x} \left[ i \right] \left[ j \right] \right) }{\sum _{i=1}^{{{\mathscr {I}}}_t}\sum _{j=1}^{\overline{{{\mathscr {B}}}}_t^{total}} chr^{x} \left[ i \right] \left[ j \right] } \end{aligned}$$

A perfect CoM for $\left( x,y \right)$ coordinate, i.e., $\left( \frac{\overline{{{\mathscr {B}}}}_{i}^{total}}{2}+\frac{1}{2} , \frac{{{\mathscr {I}}}_t}{2}+\frac{1}{2} \right)$, features a more diverse population generation. We have employed the Continuous Uniform probabilistic Distribution (CUD) for population initialization, given that the generated chromosomes satisfy the constraint. The Probabilistic distribution function of a uniform distribution over the interval $\left[ {{\mathscr {X}}}_{min}^{PHE}, {{\mathscr {X}}}_{max}^{PHE} \right]$ is given as:

14 $$\begin{aligned} f \left( {{\mathscr {X}}}_{i}^{PHE} \right) = \left\{ \begin{array}{cc} \frac{1}{{{\mathscr {X}}}_{max}^{PHE}- {{\mathscr {X}}}_{min}^{PHE}} &{} if \; {{\mathscr {X}}}_{min}^{PHE} \le {{\mathscr {X}}}_{i}^{PHE}\le {{\mathscr {X}}}_{max}^{PHE}\\ 0 &{} otherwise \end{array}\right. \end{aligned}$$

where ${{\mathscr {X}}}_{min}^{PHE}$ and ${{\mathscr {X}}}_{min}^{PHE}$ are the minimum and maximum range of the generated random variable. The mean and variance of CUD function are given as $\frac{{{\mathscr {X}}}_{min}^{PHE} + {{\mathscr {X}}}_{max}^{PHE}}{2}$ and $\frac{\left( {{\mathscr {X}}}_{max}^{PHE}- {{\mathscr {X}}}_{min}^{PHE} \right) ^{2}}{12}$, respectively.

The article "Genetic algorithm optimized node deployment in IEEE 802.15.4 potato and wheat crop monitoring infrastructure" was published in 2021. Journal: Sci Rep.

### Non-dominated shorting and crowding distance calculation

A non-dominant shorting approach begins with classifying the population ${{\mathscr {I}}}_t$ on a distant non-dominant front. A chromosome $chr^{x}[i] \mid chr^{x}[i] \in {{\mathscr {I}}}_t$ is considered a non-dominant individual if $chr^{x}[i]$ follows the relation in Eq. 15.

15 $$\begin{aligned} \begin{aligned} \lnot \; \exists \; chr^{x}\left[ i \right] \ne chr^{x}\left[ k \right] \mid \left( i,k=1,2, \cdots , {{\mathscr {I}}} \right) :&\forall j \in \left\{ 1,2,3 \right\} \left\{ {{\mathscr {O}}}^{j} \left( chr^{x}\left[ i \right] \right) \le {{\mathscr {O}}}^{j} \left( chr^{x}\left[ k \right] \right) \right\} \\&\wedge \exists \; l \in \left\{ 1,2,3 \right\} \left\{ {{\mathscr {O}}}^{l} \left( chr^{x}\left[ i \right] \right) < {{\mathscr {O}}}^{l} \left( chr^{x}\left[ k \right] \right) \right\} \end{aligned} \end{aligned}$$

The $chr^{x}[i]$ sorting operation in Eq. 15, starts with identifying all individuals on the first non-dominant front and fixes their rank by 1. Then the $chr^{x}[i]$ belonging to the second non-dominant front is identified and set to rank 2. This process continues until all fronts have been identified. To filter ${{\mathscr {I}}}$, binary tournament selection has been used. This approach randomly selects two chromosomes $chr^{x} \left[ i \right]$ and $chr^{x} \left[ j \right]$ and compares them based on rank and crowding distance. If the ranks are different, the one with the lowest rank is chosen. If they are of same rank, one with a higher crowding distance $chr^{x}_{CD}\left( i,r \right)$ is selected. The process is continued until *N* out of ${{\mathscr {I}}}$ chromosomes is selected. Initially, the crowding distance of the first and last $chr^{x}[i]$ of the front is set to infinity. For the rest of the $chr^{x}[i]$, the crowding distances $chr^{x}_{CD}$ are calculated as follow:

16 $$\begin{aligned} chr^{x}_{CD}\left( i,r \right) = \sum _{k=1}^{{{\mathscr {O}}}^{total}} \frac{\left| {{\mathscr {O}}}^{k}\left( chr^{x}\left[ i \right] +1 \right) -{{\mathscr {O}}}^{k}\left( chr^{x}\left[ i \right] -1 \right) \right| }{{{\mathscr {O}}}^{max}-{{\mathscr {O}}}^{min}} \end{aligned}$$

where *r* is the rank of the $chr^{x}[i]$, and *n* is the number of chromosome ranked *r*. The count for objective function is given by ${{\mathscr {O}}}^{total}$. Initially the crowding distance of the $chr^{x}\left[ i \right]$ is given by $chr^{x}_{CD}\left( i,r \right)$. The values ${{\mathscr {O}}}^{k}$ denotes the $k$th objective function; ${{\mathscr {O}}}^{max}$ and ${{\mathscr {O}}}^{min}$ indicate the maximum and minimum value for the objective function ${{\mathscr {O}}}^{k}$, respectively.

The article "Genetic algorithm optimized node deployment in IEEE 802.15.4 potato and wheat crop monitoring infrastructure" was published in 2021. Journal: Sci Rep.

### Crossover and mutation operation

A crossover operation combines two chromosomes to produce a new offspring. In the proposed work, chromosomes selection by crossover is based on the roulette wheel probabilities^39^. This greatly increases the likelihood of optimal solution selection and is based on fitness quality. To generate the combined solutions, a random crossover approach is applied. Which uses a single point strategy to produce two offsprings $chr^{x}_{OS}[x]$ and $chr^{x}_{OS}[y]$ by identifying a breakpoint between two chromosomes $chr^{x}[i]$ and $chr^{x}[j]$. For example, if *b* is the breaking index of the chromosomes, then the separation within two chromosomes can be represented as $chr^{x}[i] = chr^{x}[i][0 \; 1 \cdots b] + chr^{x}[i][b+1 \; b+2 \cdots \overline{{{\mathscr {B}}}}-1]$ and $chr^{x}[j] = chr^{x}[j][0 \; 1 \cdots b] + chr^{x}[j][b+1 \; b+2 \cdots \overline{{{\mathscr {B}}}}-1]$. The first half of one offspring $chr^{x}_{OS}[x]$ is taken from $chr^{x}[j]$ while the other half is taken from $chr^{x}[j]$, ie.,$chr^{x}_{OS}[x]= chr^{x}[i][0 \; 1 \cdots b] + chr^{x}[j][b+1 \; b+2 \cdots \overline{{{\mathscr {B}}}}-1]$. The composition of other offspring is: $chr^{x}_{OS}[y]= chr^{x}[i][0 \; 1 \cdots b] + chr^{x}[j][b+1 \; b+2 \cdots \overline{{{\mathscr {B}}}}-1]$. The employed mutation operation follows the bit-flip mechanism that transforms the chromosome $chr^{x}[x]$ to $chr^{x}[y] \in chr^{x}_U$ by flipping the individual bit in $chr^{x}[x]$ with probability $p=\frac{1}{\overline{{{\mathscr {B}}}}^{total}}$. Given $chr^{x}[x]$, the probability of obtaining $chr^{x}[y]$ using bit-flip mutation is given as follow:

17 $$\begin{aligned} p \left( chr^{x}\left[ x \right] \rightarrow chr^{x}\left[ y \right] \right) = p^{\left| chr^{x}\left[ x \right] \bigoplus chr^{x}\left[ y \right] \right| } \times \left( 1-p \right) ^{\overline{{{\mathscr {B}}}}^{total}-\left| chr^{x}\left[ x \right] \bigoplus chr^{x}\left[ y \right] \right| } \end{aligned}$$

The article "Genetic algorithm optimized node deployment in IEEE 802.15.4 potato and wheat crop monitoring infrastructure" was published in 2021. Journal: Sci Rep.

### Pareto-optimal solution estimation

The Pareto Optimal outcome (POS) of NSGA-II operation is a set of possible solutions ${{\mathscr {I}}}_{t}^{POS}=\left\{ chr_{POS}^{x}\left[ 1 \right] , chr_{POS}^{x}\left[ 2 \right] \cdots ,chr_{POS}^{x}\left[ z \right] \right\} \mid z=\left| {{\mathscr {I}}}_{t}^{POS} \right|$. We need to select the best solution $chr_{POS}^{x}\left[ i \right]$ from ${{\mathscr {I}}}_{t}^{POS}$ to implement $NDS^{z}$ , and hence the approach Technique for Order Performance by Similarity to Ideal Solution (TOPSIS) has been used^40^.

## Results and discussion

The proposed NSGA-II based node location optimization is performed and the chromosomes are compared over objective functions, coverage, over coverage, and RSS. A measure of the percentage of area covered and over-covered is presented to illustrate the effectiveness of individual chromosomes. A comparison with approach DT-NDS developed by Wu et al.^11^, is performed over metric RSS and coverage in target area $T^{x} \mid x \in \{wheat, potato\}$. The NSGAII-NDS outcome $(n_{i^{^{lat}}}^{x},n_{i^{^{lon}}}^{x}) \mid \forall n_{i}^{x} \in N^x$ obtained after the TOPSIS operation was employed in the target areas. The measurements were obtained for coverage and over-coverage in $T^{wheat} \mid \left| N^{wheat} \right| =25$, and are visualized by plotting $C^{wheat} [ {\overline{D}}^{T^{^{wheat}}}_{L} ] [ {\overline{D}}^{T^{^{wheat}}}_{B} ]$. The measurements for $T^{wheat}$ were collected at sowing and maturity stages, and are presented by Fig. 4a,b. Similarly, for the DT-NDS, the measurements in $T^{wheat}$ are presented in Fig. 5a,b. The RSS measurement in DT-NDS suffers more degradation than in NSGAII-NDS. Since the initial deployment in DT-NDS was done in bare land, the distance between the two nodes was more due to $\eta$ being equal to 13, and this increased the likelihood of additional RSS degradation. In the floral-initiation, terminal-spikelet-initiating and heading stages, the counter value of NSGAII-NDS is higher than DT-NDS. However, in the Grainfilling period, the DT-NDS has experienced network disconnectivity due to node isolation inception. On the other hand, $\eta$ based NSGAII-NDA strategy accounted for the possible signal degradation and outage probability threshold, resulting in a reliable IEEE 802.4.15 2.4GHz infrastructure for wheat crop monitoring.

The article "Genetic algorithm optimized node deployment in IEEE 802.15.4 potato and wheat crop monitoring infrastructure" was published in 2021. Journal: Sci Rep.

**Figure 4:** The $C^{x}[{\overline{D}}_{L}^{T^{x}}][{\overline{D}}_{B}^{T^{x}}]$ for $x=wheat$ in (**a**) sowing and (**b**) maturity stage for NSGAII-NDS. MATLAB 2016a. https://in.mathworks.com/.

**Figure 5:** The $C^{x}[{\overline{D}}_{L}^{T^{x}}][{\overline{D}}_{B}^{T^{x}}]$ for $x=wheat$ in sowing an maturity stage for GBA. MATLAB 2016a. https://in.mathworks.com/.

The wheat crop under observation is of the MP-3173 variety, which is in the category of medium height vegetation and was planted with an optimal row spacing of $22\;{\text{cm}}$. Furthermore, according to Köppen’s climate classification, the plantation location is a humid subtropical climate, with the highest and lowest temperature recorded from June 2019 to April 2020 was $49 ^{\circ }C$ and $1 ^{\circ }C$, respectively . The problem formulation and results of NSGAII-NDA may vary if the crop is grown in a different geographical area with a different variety or plantation strategy. For example, if the wheat sowing is delayed, a closer spacing of 15–18 cm is practiced, resulting in increased density per square meter. The change in density may affect the calculated path loss coefficient. To develop a comprehensive node placement strategy, path loss coefficient needs to be identified in all possible combinations of factors that can affect the receiving capability of two transceivers. Following the former goal, future works will be directed toward the collection of path loss coefficient measurements in different wheat crop varieties in different geographical regions. Furthermore, sensor nodes $n_i^x$ in WSN had a homogeneous transmission range ${{\mathscr {T}}}^x$ and could be extended to a heterogeneous ${{\mathscr {T}}}^x$ implementation. The integration of a self-adjusting ${{\mathscr {T}}}^x$ strategy into NSGAII-NDA can reduce over-coverage in the early stages of the plantation. This can be achieved by gradually increasing the ${{\mathscr {T}}}^x$ of nodes with an increase in PLC.

## Conclusion

This article proposes a reliable NSGA-II optimized Node Deployment Strategy (NDS) in the IEEE 802.15.4 wireless infrastructure for potato and wheat crop monitoring. The relationship between vegetation cover and signal attenuation for $2.4\;{\text{GHz}}$ radio frequencies has been analyzed in detail through real-time experimentation. The results of the experiment led to two significant findings; First, when the monitoring infrastructure for the wheat crop uses the NDS that was originally developed to monitor the potato crop, faces network dis-connectivity due to increased signal attenuation which is caused by growth in vegetation cover. The second finding is inferred from the first conclusion and states that it is necessary to identify a Path Loss Coefficient (PLC) in the target crop before developing NDS. The PLC has been identified at various growing stages of potato and wheat crop through empirical measurement campaigns. The implementation of the derived PLC in Lognormal path loss shadowing model was subsequently integrated into proposed NSGAII-NDS to optimize NDS over coverage, over-coverage, and Received Signal Strength (RSS). The significant difference between the NSGAII-NDS and the existing NDS strategy is that the PLC for a crop to be monitored is accounted before deployment, eliminating the possibility of a link break between two sensor nodes due to increased vegetation cover.
